# Medial Hypoxia and Adventitial Vasa Vasorum Remodeling in Human Ascending Aortic Aneurysm

**DOI:** 10.3389/fcvm.2018.00124

**Published:** 2018-09-17

**Authors:** Marie Billaud, Jennifer C. Hill, Tara D. Richards, Thomas G. Gleason, Julie A. Phillippi

**Affiliations:** ^1^Department of Cardiothoracic Surgery, University of Pittsburgh, Pittsburgh, PA, United States; ^2^McGowan Institute for Regenerative Medicine, University of Pittsburgh, Pittsburgh, PA, United States; ^3^Department of Bioengineering, University of Pittsburgh, Pittsburgh, PA, United States; ^4^Center for Vascular Remodeling and Regeneration, University of Pittsburgh, Pittsburgh, PA, United States

**Keywords:** vasa vasorum, aneurysm, hypoxia, angiogenesis, adventitia

## Abstract

Human ascending aortic aneurysms characteristically exhibit cystic medial degeneration of the aortic wall encompassing elastin degeneration, proteoglycan accumulation and smooth muscle cell loss. Most studies have focused on the aortic media and there is a limited understanding of the importance of the adventitial layer in the setting of human aneurysmal disease. We recently demonstrated that the adventitial ECM contains key angiogenic factors that are downregulated in aneurysmal aortic specimens. In this study, we investigated the adventitial microvascular network (vasa vasorum) of aneurysmal aortic specimens of different etiology and hypothesized that the vasa vasorum is disrupted in patients with ascending aortic aneurysm. Morphometric analyses of hematoxylin and eosin-stained human aortic cross-sections revealed evidence of vasa vasorum remodeling in aneurysmal specimens, including reduced density of vessels, increased lumen area and thickening of smooth muscle actin-positive layers. These alterations were inconsistently observed in specimens of bicuspid aortic valve (BAV)-associated aortopathy, while vasa vasorum remodeling was typically observed in aneurysms arising in patients with the morphologically normal tricuspid aortic valve (TAV). Gene expression of hypoxia-inducible factor 1α and its downstream targets, metallothionein 1A and the pro-angiogenic factor vascular endothelial growth factor, were down-regulated in the adventitia of aneurysmal specimens when compared with non-aneurysmal specimens, while the level of the anti-angiogenic factor thrombospondin-1 was elevated. Immunodetection of glucose transporter 1 (GLUT1), a marker of chronic tissue hypoxia, was minimal in non-aneurysmal medial specimens, and locally accumulated within regions of elastin degeneration, particularly in TAV-associated aneurysms. Quantification of GLUT1 revealed elevated levels in the aortic media of TAV-associated aneurysms when compared to non-aneurysmal counterparts. We detected evidence of chronic inflammation as infiltration of lymphoplasmacytic cells in aneurysmal specimens, with a higher prevalence of lymphoplasmacytic infiltrates in aneurysmal specimens from patients with TAV compared to that of patients with BAV. These data highlight differences in vasa vasorum remodeling and associated medial chronic hypoxia markers between aneurysms of different etiology. These aberrations could contribute to malnourishment of the aortic media and could conceivably participate in the pathogenesis of thoracic aortic aneurysm.

## Introduction

The tunica adventitia of large blood vessels includes extracellular matrix and diverse cell types constituting a unique microenvironment distinct from the neighboring tunica media. In elastic conduit arteries, this outer layer provides substantial biomechanical support and is thought to be critically important in maintaining vascular homeostasis (1, 2). However, the biological mechanisms by which the adventitia influences large blood vessels' functions are less understood. Despite this gap in knowledge, a growing body of evidence supports a critical role for adventitia in vascular wall physiology and pathophysiology (3–6).

In addition to luminal flow, large blood vessels require their own external access to a blood supply to maintain vascular health. The *vasa vasorum* (Latin: “vessels of the vessels”) serves this vital role in large blood vessels. During his research on anatomy in the seventeenth century, Willis was purportedly the first to report the existence of vasa vasorum in the aorta (7). Since this first acquaintance, the purpose and functionality of this extensive microvascular network have barely begun to be understood. In human, the ascending thoracic aorta has an expansive network of vasa vasorum that originates from the coronary and brachiocephalic arteries (7, 8). The vasa vasorum infiltrates the blood vessel wall from the abluminal side and weaves extensively through the adventitial layer. The arteries of the vasa vasorum supply oxygen and nutrients to the outer two-thirds of larger blood vessels (>0.5 mm thick) comprised of at least 29 elastic lamellae at birth (e.g., thoracic aorta, pulmonary artery, and saphenous vein of humans, sheep and dogs) while the veins remove waste products (9, 10). Blood vessels with fewer than 29 elastic lamellae, with the exception of coronary arteries or certain disease states, are devoid of vasa vasorum in the outer media such as those of small rodents, and are adequately nourished from the lumen (9). Nearly half a century ago, the importance of the vasa vasorum was realized from observations of ischemic medial necrosis in the canine ascending aorta following occlusion of the vasa vasorum (11). Other investigators have reproduced these findings in other animal models and corroborated the remodeling of the aortic wall, which is reminiscent of the histopathological hallmark of cystic medial degeneration in human thoracic aortic aneurysm (10, 12–14). These studies raised important questions on the role of the vasa vasorum in human aortic disease.

Our laboratory focuses on ascending thoracic aortic aneurysm (TAA), the main pathology known to affect the ascending aorta. TAAs can arise in patients with the morphologically normal tricuspid aortic valve (TAV), but patients with the most common congenital anomaly of the aortic valve (bicuspid aortic valve, BAV) have a heightened risk of developing aneurysm in the proximal ascending aorta (15, 16). Our work has centered on understanding the cellular and molecular mechanisms involved in TAAs arising in both patient populations (17–20). We have uncovered mechanisms distinctly involved in BAV aortopathy, such as altered response to oxidative stress (17), unique medial matrix architecture (21), and altered biomechanical strength (22). Considering these findings mostly focused on the aortic media, we extended our interests to the adventitia as an important neighboring microenvironment in the setting of aortic disease. We concentrated on the vasa vasorum network specifically and hypothesized that this microvascular network is disrupted in patients with TAA. Here, we describe remodeling of vasa vasorum vessels and note aberrations in size, abundance and wall thickness in TAA specimens associated with down-regulation of angiogenic and hypoxia-related gene targets in the adventitial layer while the medial layer displayed evidence of hypoxia. These aberrations uncover a new view of the pathophysiology of human thoracic aortic disease from the perspective of the adventitia.

## Materials and methods

### Tissue collection and processing

Human ascending thoracic aortic specimens (*n* = 91) were collected during elective aortic valve and ascending aortic replacement operations or during heart transplantation with informed patient consent and approval of the Institutional Review Board of the University of Pittsburgh and through the Center for Organ Recovery and Education. All patient-related procedures were carried out in accordance with principles outlined in the Declaration of Helsinki. The aortic specimens were obtained within 1–2 cm of the sinotubular junction. Upon excision, tissue specimens were placed in saline on ice and transported to the laboratory. Specimens were categorized according to their aortic valve morphology: tricuspid (TAV) or bicuspid (BAV). Patient demographics, aortic dimensions, and comorbidities, (e.g., hypertension) were carefully recorded (Table 1). None of the included patients had diagnosed Marfan, Ehlers-Danlos or Loeys-Dietz syndromes or chronic or acute dissection. Patients are otherwise relatively healthy. Maximal orthogonal aortic diameter was measured via intraoperative trans-esophageal echocardiography. The non-aneurysmal cohorts included patients with maximal orthogonal diameters of ≤ 42 mm. The aneurysmal patient cohorts included patients undergoing ascending aortic replacement due to ascending TAA and exhibited a maximal orthogonal aortic diameter >42 mm.

**Table 1:** Patient demographics.

	**TAV**		**BAV**	
	**NA**	**TAA**	**NA**	**TAA**
*N* (M/F)	40 (23/16)^a^	39 (22/17)	31 (20/11)	44 (35/9)
Age (year)	56 ± 16.9	67 ± 8.7*	57 ± 11.2^∧^	56 ± 10.6^∧^
Diameter (mm)	32 ± 3.4^b^	52 ± 5.8*	38 ± 3.8^c^	51 ± 3.9*^∧^
AI 1+	5.3%	23.1%	16.7%	20.9%
2–3+	15.8%	35.9%	6.7%^∧^	18.6%
4+	5.3%	20.5%	26.9%	11.6%
AS Mild	0%	0%	0%	23.1%^∧#^
Mod	0%	0%	3.3%	15.4%^∧#^
Severe	25.0%	7.7%	76.7%^*∧^	30.7%^∧#^
HTN	50.0%	76.9%*	61.3%	70.5%
Diabetes	17.5%	13.5%	12.9%	23.3%
Smoking	47.5%	43.2%	43.4%	45.5%
ARB	0%	17.9%*	38.7%^*∧^	9.1%^*∧^
ACE-inhibitor	35%	10.8%*	12.1%	37.2%^∧#^
Statins	27.5%	53.8%*	64.5%*	43.2%*

*Quantitative data are presented as median ± SD*.

*, #, and ∧ indicate significance vs. TAV-NA, BAV-NA, and TAV-TAA, respectively and were obtained using a Chi-squared or a Kruskal-Wallis test.

*HTN, hypertension; S.D., standard deviation; ARB, angiotensin-receptor blocker; ACE, angiotensin-converting enzyme; AS, aortic stenosis, AI, aortic insufficiency*.

a *Sex of one patient was not recorded*.

b,c *Calculated from data from 17 and 22 patients, respectively*.

### Histology and immunofluorescence

Portions (~0.5 cm^2^) of human aortic specimens were fixed in 10% buffered formalin overnight or 4% paraformaldehyde for 30 min and paraffin-embedded. Cross-sections (5 μm) were stained with hematoxylin and eosin (H&E) to reveal aortic layers and vasa vasorum structures (McGowan Institute for Regenerative Medicine Histology Core, University of Pittsburgh). Sections were reviewed by two authors (MB and JP). Before immunolabeling, paraffin was removed using xylene followed by an ethanol dehydration series, rehydration in water and phosphate buffer saline (PBS) and antigen retrieval (Target Retrieval Solution, pH 6, Dako #S1700). Blocked slides (0.5% bovine serum albumin) were incubated in primary un-conjugated antibody (α-SMA, 1:1000, DAKO, # M0851, GLUT1, 1:500, Millipore #07-1401) in blocking solution overnight at 4°C. Secondary labeling was accomplished with Alexa Fluor-conjugated secondary antibodies (anti-mouse Alexa Fluor 594, # 715-585-150, anti-rabbit Alexa Fluor 594, # 711-585-152, all from Jackson Immunoresearch) for 2 h at room temperature. A FITC-conjugated antibody targeting Von Willebrand Factor was added to the secondary labeling step (1:100, US Biological, # V2700-01C). Sections were mounted with coverslips using Prolong Gold with DAPI (Invitrogen, # P-36931) and allowed to dry overnight. Slides were visualized using a TE-2000-E inverted microscope (Nikon) using bright field or epi-fluorescence microscopy and captured using a DS-Fi1 5MP color camera (Nikon) or an Imaging Array CoolSNAP ES2 Monochrome 1,394 × 1,040 High Resolution Camera (Photometrics) and NIS Elements Software 3.2 (Nikon). Vasa vasorum morphometrics were independently calculated from the entirety of each section using NIS Elements Software by two researchers (MB and JP) and similar outcomes were observed for each. Reported vessel diameters and lumen areas were calculated from vessel perimeter measurements. Vessel thickness was calculated by normalizing the vessel wall area to the lumen diameter. Vasa vasorum density was calculated from the total number of vessels observed on aortic cross sections and divided by the adventitial area. To limit the influence of potential histological embedding and sectioning artifacts, a binary thresholding method was employed to quantify adventitial tissue area. Inflammatory infiltrates were described by a clinical pathologist of the University of Pittsburgh Medical Center.

### RNA isolation and quantitative real-time PCR

Portions of aortic adventitial specimens were swiftly placed in RNA*later* solution (Life Technologies) and stored at −20°C until use. Specimens (15–20 mg) were homogenized in RLT buffer (QIAgen) containing β-mercaptoethanol (1/100, Fisher Scientific BP176-100) using the gentleMACS Tissue Dissociator (Miltenyi, Auburn, CA). Further homogenization was achieved using the QIAshredder kit (Qiagen). Total RNA was isolated from adventitial tissue extracts using the RNAeasy Plus Mini kit (QIAgen) according to the manufacturer's instructions. Gene expression of hypoxia-inducible factor 1 alpha (*Hif-1*α), vascular endothelial growth factor (*Vegf*), and metallothionein (*Mt*)-1A were quantified from 5 to 25 ng of template RNA using inventoried Taqman® Gene Expression Assays and 1-step RNA-to-CT™ kit (Life Technologies). Primer set details can be found in Table 2. Thermocycling conditions were as follows: RNA was reverse-transcribed at 48°C for 15 min followed by *Taq* activation at 95°C for 10 min, and 40 cycles of denaturation for 15 s at 95°C, and primer and probe annealing at 60°C for 1 min. All target gene probes were labeled with FAM as the 5′ reporter dye and TAMRA as the 3′ quencher dye. Assays were carried out in triplicate on an ABI Prism 7900HT sequence detection system in the Genomics and Proteomics Core Laboratories of the University of Pittsburgh. Data was analyzed using SDS 2.2.2 Software (Applied Biosystems). Relative gene expression levels were calculated using the ΔC_T_ and reported as relative gene expression normalized to *PPIA* as the endogenous control.

**Table 2:** Primer set details.

**Gene name**	**Gene symbol**	**Assay ID #**
Hypoxia-inducible factor 1α	*Hif-1α*	Hs00936366_m1
Metallothionein IA	*Mt-1A*	Hs00831826_s1
Vascular endothelial growth factor	*Vegf-A*	Hs00900055_m1

### Western blotting

Ascending aortic media specimens were mechanically processed to remove the adventitial and the intimal layers. The resulting aortic medial specimens were homogenized in RIPA buffer (Pierce) containing phosphatase and protease inhibitor cocktails (ThermoFisher and Sigma, respectively) and phenylmethanesulfonylfluoride (PMSF, Sigma) using the gentleMACS Tissue Dissociator. Following a low-speed centrifugation (1,500 g for 5 min at 4°C), samples were placed on ice for 30 min. Samples were then centrifuged at high speed (12,000 g) for 20 min at 4°C and protein concentration of the supernatant was determined using the bicinchoninic acid (BCA) assay (Pierce).

Western blotting was performed using standard procedure as previously described (18). Briefly, samples were mixed with Laemmli buffer and boiled at 100°C for 5 min. Electrophoresis was performed on SDS-PAGE containing 10% acrylamide and proteins were transferred to polyvinylidene fluoride membrane. After blocking for 1 h in blotting-grade blocker (BioRad), membranes were incubated overnight at 4°C with an anti-GLUT1 antibody (1:500, Millipore #07-1401), rinsed in PBS-Tween-20 0.1% and incubated for 2 h at room temperature with an anti-goat antibody coupled to horseradish peroxidase (Santa Cruz Biotechnology, #sc-2020). Protein bands were visualized using enhanced chemiluminescence Western Blotting Substrate (Pierce), captured using a ChemiDoc imager (BioRad) and quantified using ImageLab software (BioRad). Membranes were stripped in Re-Blot Plus Strong Solution (EMD Millipore) and re-probed with an anti-β-actin antibody (1:5,000, Abcam, #ab8227) for normalization. Relative GLUT1 expression was calculated as the ratio of Glut1 band density over β-actin band density for each sample.

### Thrombospondin-1 ELISA

Aortic adventitial specimens were placed in RIPA buffer supplemented with protease and phosphatase inhibitors and protein lysates were prepared as described above for aortic medial samples. The BCA assay was employed to determine the protein concentration of each sample and 25 μg of adventitial lysates were used to determined TSP1 levels via ELISA following the manufacturer's instructions (R&D).

### Statistical analyses

Quantitative data are reported in the text as mean ± standard error of the mean and are represented in figures in hanging box plot format, where median and interquartile ranges are shown, and error bars represent 90 and 10th percentile (SigmaPlot 12.5). Outliers were excluded using the Outlier Labeling Rule according to Hoaglin and Iglewicz (23) and using SPSS Statistic software version 24.0 (IBM Corp.) Prevalence of hypertension, aortic stenosis and aortic insufficiency were compared between patient groups using a Chi-Squared test. All other data were compared using the non-parametric Mann-Whitney test or the Kruskal-Wallis followed by a Dunn's *post-hoc* test, as indicated in each figure legend. A *p*-value of < 0.05 was considered significant. When indicated, variables were evaluated for correlation using the bivariate Pearson correlation analysis.

## Results

### Decreased density of vasa vasorum in thoracic aortic aneurysm

We histologically evaluated the adventitia of aneurysmal aortic specimens and examined the abundance of vasa vasorum in comparison to their non-aneurysmal counterparts (Figures 1A–H). Inspection of H&E stained aortic cross sections revealed less density of vessels in aneurysmal TAV patients when compared with non-aneurysmal aortas from TAV patients (11.9 ± 1.53 vs. 24.7 ± 3.04 vessels/mm^2^, respectively, *p* = 0.004, Figure 1I). The density of vasa vasorum in aneurysmal and non-aneurysmal BAV specimens was similar to that of non-aneurysmal TAV specimens (19.8 ± 2.45 and 24.7 ± 3.26 vs. 24.7 ± 3.04 vessels/mm^2^, *p* = 0.224 and *p* = 0.922, respectively, Figure 1I). Interestingly, when data from aneurysmal BAV and TAV specimens were compared, the density of vasa vasorum was higher in aneurysmal BAV specimens (19.8 ± 2.45 vs. 11.9 ± 1.53 vessels/mm^2^, *p* = 0.009). Of note, when normalized to the total section area, we found that the adventitial area was larger in aneurysmal specimens when compared to non-aneurysmal specimens (11.1 ± 1.0 vs. 8.1 ± 0.8% of total section area, *p* = 0.002). Normalized adventitial area was highest in TAV-TAA specimens when compared to all other groups (14.7 ± 1.7 vs. 7.8 ± 1.2 (TAV-NA), 8.6 ± 1.1% (BAV-NA) and 9.6 ± 0.8% (BAV-TAA), *p* < 0.02). Analysis of vasa vasorum density as a function of the ascending aortic diameter revealed a negative correlation in specimens from TAV patients only (Pearson's ρ = −0.544, *p* = 0.002, Figure 1J). There was no correlation between vasa vasorum density and aortic diameter in specimens from BAV patients (*p* = 0.913, Figure 1H). There was no correlation of vasa vasorum density with age of the patients.

**Figure 1:** Reduced vasa vasorum density in human ascending aortic adventitia of aneurysmal TAV patients. Representative H&E staining of specimens from a non-aneurysmal (NA) patient with a morphologically normal tricuspid aortic valve (TAV) **(A, B)** or with a bicuspid aortic valve (BAV) **(C, D)**. Images in **(E,F)** show representative H&E staining of aneurysmal (TAA) specimens from a TAV patient and in **(G,H)**, from a BAV patient. Images in **(A,C,E,G)** depict an aortic specimen that were captured with a 20X objective and tiled to comprise the entire section, scale bar = 500 μm. Panels **(B**,**D**,**F,H)** represent magnification of insets denoted in the corresponding image in the left panel and are representative of the observed reduced density of vasa vasorum (arrows) in aneurysmal specimens. Images were captured with a 20X objective, scale bar = 50 μm. Images of vasa vasorum in the adventitia (adv) were captured adjacent to the tunica media (med). Dashed line = adv-med border. **(I)** Quantification of vessel density as number of vessels per mm^2^ of adventitia. * and ^∧^ indicates *p* < 0.05 vs. TAV-NA and TAV-TAA, respectively and assessed with the Kruskal-Wallis test. **(J)** Graphical representation of vessel density as a function of the maximal orthogonal aortic diameter (MOAD) in TAV (red) and BAV (blue) specimens. ρ indicates the coefficient of correlation and *p* indicates the *p*-value obtained using a bivariate Pearson correlation analysis.

### Increased vasa vasorum lumen size in thoracic aortic aneurysm

Inspection of the vessel size revealed increased lumen area in aneurysmal aortas from BAV patients compared to specimens from non-aneurysmal BAV patients (1,338 ± 230 vs. 691 ± 126 mm^2^, *p* = 0.022, Figures 2A–E). However, the lumen area in aneurysmal TAV and BAV patients was similar when compared to non-aneurysmal TAV specimens (1,093 ± 174 mm^2^ and 1,338 ± 230 vs. 866 ± 132 mm^2^, *p* = 0.329 and *p* = 0.128, respectively, Figure 2E). The lumen area of all aneurysmal specimens (BAV and TAV combined) were collectively larger than the lumen area of all the non-aneurysmal specimens combined (1,524 ± 263 vs. 789 ± 92.3, *p* = 0.013, Figure 2E). While there was no correlation found between lumen area of vasa vasorum and patients' age for TAV or BAV cohorts, the lumen area was positively correlated with maximal orthogonal aortic diameter in BAV specimens only (Pearson's ρ = 0.351, *p* = 0.036, Figure 2F).

**Figure 2:** Increased vasa vasorum lumen area in human ascending aortic adventitia of aneurysmal patients. Representative images of aortic specimens stained with H&E collected from non-aneurysmal (NA) or aneurysmal (TAA) patients with a morphologically normal tricuspid aortic valve (TAV) **(A,C)** or with a bicuspid aortic valve (BAV) **(B,D)**. Specimens were imaged with a 20X objective, scale bar = 50 μm. The border between the adventitia (adv) and the media (med) is denoted by a dashed line. Quantification of vasa vasorum lumen area (mm^2^) in the four patient cohorts is shown in **(E)**. # indicates *p* < 0.05 vs. BAV-NA and was obtained using a Kruskal-Wallis test. The *p*-value indicated above the graph was determined using a Mann-Whitney test comparing data collected in all aneurysmal specimens to those collected in all non-aneurysmal specimens. Vessel density was expressed as a function of the maximal orthogonal aortic diameter (MOAD) in TAV (red) and BAV (blue) specimens **(F)**. ρ indicates the coefficient of correlation and *p* indicates the *p*-value obtained using a bivariate Pearson correlation analysis.

We further compared the relative distribution of vessel size according to the classification described by Giannoni et al. (24). Aneurysmal aortic specimens from both TAV and BAV patients displayed less small vessels (lumen diameter < 50 μm) when compared to non-aneurysmal TAV specimens (8.49 ± 1.17 and 10.6 ± 1.41 vs. 19.6 ± 2.55, *p* < 0.001 and *p* = 0.005, respectively, Figure 3A). The density of small size vessels was also lower in aneurysmal BAV specimens when compared to that of non-aneurysmal BAV specimens (10.6 ± 1.41 vs. 19.3 ± 2.79, *p* = 0.022, Figure 3A). With respect to mid-size vessels (50–100 μm), their density was lower in aneurysmal TAV specimens when compared to non-aneurysmal TAV specimens (1.26 ± 0.16 vs. 5.12 ± 1.14, *p* = 0.037, Figure 3B). In contrast, aneurysmal BAV specimens displayed a similar density of mid-size vessels when compared to non-aneurysmal BAV specimens (3.50 ± 0.47 vs. 3.93 ± 0.64, *p* = 0.929, Figure 3B), but a higher number of mid-size vessels were observed when compared to aneurysmal TAV specimens (3.50 ± 0.47 vs. 1.26 ± 0.16, *p* = 0.027, Figure 3B). Quantification of large vasa vasorum (>100 μm of diameter) showed that all aneurysmal specimens displayed more numerous large vasa vasorum when compared to all non-aneurysmal specimens (1.79 ± 0.24 vs. 1.16 ± 0.25, *p* = 0.028, Figure 3C). We identified negative correlations between small vessel density and ascending aortic diameter in both BAV- and TAV-associated aortopathy (ρ = −0.358, *p* = 0.038 for BAV specimens and ρ = −0.526, *p* = 0.003 for TAV specimens Figure 3D). While mid-size density was negatively correlated with ascending aortic diameter in TAV specimens (ρ = −0.407, *p* = 0.023, Figure 3E), there was no correlation between large size vessels and ascending aortic diameter. Conversely, mid-size vessels displayed no correlation with ascending aortic diameter in BAV specimens, while the density of large vessels increased with ascending aortic diameter (ρ = 0.357, *p* = 0.035, Figure 3F). Pearson's correlation tests on the density of the different sizes of vasa vasorum and age of the patients were not significant.

**Figure 3:** Aneurysmal specimens are characterized by a lower density of small size vasa vasorum. **(A–C)** Quantification of small size (< 50 μm, **A**), mid-size (50–100 μm, **B**) and large (>100 μm, **C**) vasa vasorum density as number of vessels per mm^2^ of adventitia. *, #, and ^∧^ indicate *p* < 0.05 vs. TAV-NA, BAV-NA, and TAV-TAA, respectively and were obtained using a Kruskal-Wallis test. The *p*-value indicated above the graph in **(C)** was obtained using a Mann-Whitney test comparing data collected in all aneurysmal specimens to those collected in all non-aneurysmal specimens. **(D–F)** Graphical representation of small **(D)**, mid-size **(E)**, and large **(F)** vessel density as a function of the maximal orthogonal aortic diameter (MOAD) in TAV (red) and BAV (blue) patients. ρ indicates the coefficient of correlation and *p* indicates the *p*-value obtained using a bivariate Pearson correlation analysis.

### Vasa vasorum wall remodeling in thoracic aortic aneurysm

Qualitative inspection of vasa vasorum structures revealed disparity in the thickness of the vessel wall (Figures 4A–D). Immunolabeling revealed more numerous α-SMA positive and vWF negative cells in the thickened vasa vasorum walls (Figures 4E–H). Measurement of vasa vasorum wall area normalized to the lumen diameter revealed increased vessel wall thickness in aneurysmal TAV aorta when compared with non-aneurysmal TAV aorta (52.8 ± 4.39 vs. 37.0 ± 3.83, *p* = 0.07, Figure 5A). The vasa vasorum wall thickness was similar among all non-aneurysmal specimens and aneurysmal BAV specimens, and aneurysmal BAV specimens displayed less thick vasa vasorum when compared to aneurysmal TAV specimens (40.5 ± 5.28 vs. 52.8 ± 4.39, *p* = 0.031). Comparison of vasa vasorum thickness and ascending aortic diameter revealed a positive correlation between the two variables in TAV specimens only (ρ = 0.393, *p* = 0.026, Figure 5B). The vasa vasorum thickness was not correlated with age of the patients.

**Figure 4:** Vasa vasorum in the adventitia of TAV-TAA specimens display smooth muscle remodeling. **(A–D)** H&E stained sections of non-aneurysmal (NA, **A,B**) and aneurysmal (TAA, **C,D**) specimens isolated from patients with TAV **(A,C)** or BAV **(B,D)**. **(E–H)** Immunolabeling for α-SMA (red), Von Willebrand factor (vWF, green), and nuclei (DAPI, blue) performed on vessels displayed in A through D. All images were obtained with a 40X objective, scale bar = 50 μm.

**Figure 5:** Vasa vasorum wall thickening in the adventitia of TAV-TAA patients. **(A)** Quantification of vasa vasorum smooth muscle area from H&E stained sections and normalized to lumen diameter. * and ^∧^ indicate *p* < 0.05 vs. TAV-NA and TAV-TAA, respectively and were obtained using a Kruskal-Wallis test. **(B)** Graphical representation of the vasa vasorum wall thickness as a function of the maximal orthogonal aortic diameter (MOAD) in TAV (red) and BAV (blue) specimens. ρ indicates the coefficient of correlation and *p* indicates the *p*-value obtained using a bivariate Pearson correlation analysis.

### Decreased expression of pro-angiogenic and hypoxia gene targets in the adventitia of aneurysmal patients

To investigate possible reasons for altered vasa vasorum density, we examined expression of gene targets associated with angiogenic and hypoxic signaling. Real-time PCR experiments on total mRNA from adventitial specimens revealed that expression of *hypoxia-inducible factor-1 alpha* (*Hif-1*α*)* was down-regulated in adventitial specimens from aneurysmal BAV specimens when compared with specimens from non-aneurysmal TAV and BAV specimens (0.022 ± 0.005 vs. 0.069 ± 0.018, *p* = 0.008, and vs. 0.041 ± 0.006, *p* = 0.037, Figure 6A). Down-regulation of *Hif-1*α downstream gene targets *vascular endothelial growth factor (Vegf)* and *metallothionein* (*Mt-1A)* was also noted in the adventitia of aneurysmal specimens when compared with non-aneurysmal specimens TAV patients (0.024 ± 0.003 vs. 0.059 ± 0.014, *p* = 0.049, Figure 6B and 0.0077 ± 0.0015 vs. 0.048 ± 0.016, *p* = 0.018, Figure 6C). Additionally, the adventitia of BAV-TAA specimens contained lower amounts of *Mt-1A* mRNA in comparison to TAV-NA specimens (0.0109 ± 0.0016 vs. 0.048 ± 0.016, *p* = 0.046, Figure 6C). When gene expression from all aneurysmal specimens was compared to all non-aneurysmal specimens, *Hif-1*α and *Mt-1A* expression level were found to be lower (0.028 ± 0.004 vs. 0.055 ± 0.010, *p* = 0.013, Figure 6A and 0.033 ± 0.008 vs. 0.009 ± 0.001, *p* = 0.019, Figure 6C). Protein expression level of the anti-angiogenic factor thrombospondin-1 (TSP1) was elevated in TAV-TAA specimens when compared to TAV-NA specimens (227 ± 67 vs. 62 ± 14 ng/ml, *p* = 0.022, Figure 6D). Lastly, all aneurysmal specimens contained higher amounts of TSP1 when compared to all non-aneurysmal specimens (183 ± 40 vs. 81 ± 14 ng/ml, *p* = 0.038, Figure 6D).

**Figure 6:** Expression of angiogenesis and hypoxia-related target genes in human ascending aortic adventitia. Quantitative real-time PCR was employed to measure expression of *Hif-1*α **(A)**, *Vegf-A* **(B)** and *Mt-1A* **(C)** in total mRNA isolated from adventitia of human ascending aortic specimens. Thrombospondin 1 (TSP1) levels were quantified via ELISA in 25 μg of adventitial lysates **(D)**. * and # indicate *p* < 0.05 vs. TAV-NA and BAV-NA, respectively and were obtained using a Kruskal-Wallis test. The *p*-values indicated above the graphs were obtained using a Mann-Whitney test comparing data collected in all aneurysmal specimens to those collected in all non-aneurysmal specimens.

### Chronic hypoxia in the media of aneurysmal specimens

To explore the potential effects of adventitial vasa vasorum remodeling on the aortic media, we probed for evidence of chronic hypoxia using immuno-based detection of the glucose transporter GLUT1 (Figure 7). We found that GLUT1 was abundantly present within the aortic media of aneurysmal specimens and primarily localized to areas of elastin degeneration in TAV-TAA specimens (Figure 7A). In contrast, qualitative inspection of non-aneurysmal aortic media revealed visibly lower levels of GLUT1 expression. Quantification of GLUT1 expression in lysates of aortic media specimens confirmed elevated levels of expression in aneurysmal aorta when compared to non-aneurysmal aorta for specimens from patients with TAV (1.08 ± 0.16 vs. 0.58 ± 0.08, *p* = 0.006, Figure 7B). Similarly, aneurysmal aortic specimens from BAV patients exhibited increased GLUT1 protein expression when compared to non-aneurysmal specimens from patients with TAV (0.99 ± 0.12 vs. 0.58 ± 0.08, *p* = 0.011, Figure 7B). GLUT1 expression was higher in all aneurysmal specimens when compared with all non-aneurysmal specimens (1.04 ± 0.10 vs. 0.66 ± 0.06, *p* = 0.004). Expression levels of Glut1 were positively correlated with ascending aortic diameter in TAV specimens only (ρ = 0.513, *p* = 0.036, Figure 7C).

**Figure 7:** Detection of glucose transporter 1 (GLUT1) in the aortic media. **(A)** GLUT1 expression (red) was assessed via immunofluorescence on aortic cross section of aneurysmal and non-aneurysmal specimens excised from patients with TAV (top row) or BAV (bottom row). The elastin autofluorescence appears in green and DAPI-stained nuclei are shown in blue. Scale bar = 50 μm. **(B)** Quantification of GLUT1 expression via western blot on aortic media lysates of non-aneurysmal (NA) and aneurysmal (TAA) specimens from TAV and BAV patients. The intensity of the band corresponding to GLUT1 (54 kDa) was normalized to that of β-actin. * indicates *p* < 0.05 vs. TAV-NA and was obtained using a Kruskal-Wallis test. The *p*-value indicated above the graphs was obtained using a Mann-Whitney test comparing data collected in all aneurysmal specimens to those collected in all non-aneurysmal specimens. **(C)** Graphical representation of GLUT1 expression levels as a function of the maximal orthogonal aortic diameter (MOAD) in TAV (red) and BAV (blue) specimens. ρ indicates the coefficient of correlation and *p* denotes the *p*-value obtained using a bivariate Pearson correlation analysis.

### Adventitial inflammation in specimens of degenerative thoracic aortic aneurysm

While there was no evidence of an inflammatory infiltrate in specimens from non-aneurysmal patients (Figures 8A,B), we noted an extensive chronic inflammatory component in the adventitia of aneurysmal patients. Evidence of a lymphoplasmacytic infiltrate was found in the majority of aneurysmal specimens from patients with TAV (92%, Figures 8C,D) and was observed only in 25% of aneurysmal specimens from patients with BAV (Figures 8E,F). Images representative of specimens from aneurysmal TAV patients (Figures 8C,D) and BAV patients (Figures 8E,F) reveal infiltration of lymphocytes and plasma cells (arrowheads) localized to smaller vessels of the vasa vasorum within the adventitia.

**Figure 8:** Chronic inflammation in the ascending aortic adventitia of aneurysmal specimens. **(A,B)** Representative H&E staining of TAV-NA and BAV-NA, respectively where no inflammatory infiltrate was found. **(C,D)** Representative H&E staining of TAV-TAA and BAV-TAA exhibiting lymphoplasmacytic infiltration localized to small diameter vasa vasorum. Plasma cells are marked by arrowheads. These findings were more prevalent in specimens isolated from aneurysmal patients with TAV **(E)** and mostly absent from aneurysmal specimens of patients with BAV **(F)**. Scale bar = 25 μm.

## Discussion

In large vessels such as the aorta, blood perfusion from the aortic lumen is the principal source of nutrients and oxygen for the cells located on the luminal side, while the vasa vasorum provides nourishment to cells located on the abluminal side (25, 26). Specifically, work in animals uncovered that this microvascular network supplies the adventitia and the smooth muscle cells located in the outer third of the medial layer with oxygen and nutrients (10). Because medial degeneration, which includes loss of smooth muscle cells, is characteristic of ascending aortic aneurysms, we reasoned that alterations in the adventitial vasa vasorum network may play a role in aneurysm pathophysiology. In support of this concept, we reveal adventitial vasa vasorum remodeling and down-regulation of angiogenic signaling in the adventitia of specimens of human ascending aortic aneurysm, along with evidence of chronic hypoxia in the medial layer.

In our study of human aortic specimens, the decreased density of vasa vasorum and their significant remodeling in TAA, along with the altered distribution of vessel size could all lead to reduced blood flow to the medial layer. While our findings of increased lumen area of the vasa vasorum might be presumed to deliver a larger blood volume, a “paradoxical decrease” in blood flow through a dilated vasa vasorum has been documented following angioplasty in the canine (27). Nevertheless, our results reveal evidence of chronic hypoxia in the media with increased expression levels of GLUT1, a gene target of HIF1α (28). Increased expression of GLUT1 occurs during anaerobic glycolysis and is indicative of a state of chronic hypoxia. Our results are suggestive of a chronic hypoxic environment in the media of aneurysmal ascending aortic specimens alongside intense remodeling of vasa vasorum in the neighboring adventitia. A recent study by Niinimaki et al. corroborates this notion, since the authors described higher expression of another player in the hypoxic pathway, carbonic anhydrase IX, in the media of aneurysmal ascending aortic specimens (29). The adventitia of aneurysmal specimens coincided with down-regulation of hypoxia-related genes, including *Hif-1*α and its signaling targets *Vegf* and *Mt1a*. Interestingly, we previously demonstrated reduced levels of *Mt-1a* gene expression, while *Vegf* gene expression was unchanged in the media of aneurysmal ascending aortic specimens from BAV patients compared to that of non-aneurysmal patients with TAV (17, 30). Although hypoxia-triggered signaling typically involves post-translational activation of HIF-1α and induction of downstream targets, including *Mt-1a* (31) and *Vegf* (32), chronic local tissue hypoxia has been shown to decrease VEGF signaling and angiogenic response via a HIF1α-dependent mechanism in human endothelial cells (33). Furthermore, since MT has been shown to rescue HIF-1α transcriptional activity in other systems (34), the reduction of *Mt-1A* in the adventitia could further limit transcription of hypoxia gene targets such as *Vegf* as we demonstrated here. This theory of hypoxia-mediated down-regulation of VEGF signaling agrees with our observation of a less dense vasa vasorum network and less small vessels (< 50 μm) in the adventitia of aneurysmal specimens. Taken together, down-regulation of key gene targets of angiogenesis and hypoxic signaling in the adventitia of aneurysmal thoracic aorta might be a consequence of the chronic hypoxia in the media and could have been initially triggered by reduced perfusion of the adventitia due to alterations in the vasa vasorum network. These findings collectively underscore the complexity of thoracic aortic disease and additional studies will address how adventitial hypoperfusion relates to medial hypoxia.

Our findings of thickened walls of vasa vasorum in the adventitia of aneurysmal aortic specimens agree with those reported by Osada et al. who described evidence of intimal sclerotic thickening in dissected human aorta (35). Furthermore, TAA arising in patients with mutations in the genes encoding the smooth muscle cytoskeletal proteins *Acta2* and *Myh11* also displayed local SMC hyperplasia and occlusion of the vasa vasorum (36, 37). While hyperplastic thickening of the vasa vasorum has been reported in cases of syphilitic aortitis, causing restricted blood flow to the media with resultant ischemia (38), none of the patients in our study had a history of syphilis. Rather, the vasa vasorum thickening noted in our study was presumably due to outward remodeling of their smooth muscle layer, which is likely to be associated with alterations of the vasa vasorum contractility. In the healthy aortic wall, blood flow regulation in the vasa vasorum network is complex. While sympathetic innervation contributes to adventitial blood flow regulation, vasa vasorum react to several contractile and dilatory agonists *ex vivo* (39, 40). The effect of microvessel thickening and smooth muscle hyperplasia on vasa vasorum contractility and blood flow regulation warrant further considerations in the context of aortic diseases.

Despite a few observations in aneurysmal diseases, the contribution of vasa vasorum in diseases of large vessels has been primarily examined in the setting of atherosclerosis, where multiple inflammatory pathways drive vasa vasorum expansion from the adventitia to the neointima (26). These inflammatory pathways are thought to be stimulated by an increase in oxygen demand as the wall thickness of the diseased vessel increases and consequently leads to hypoxia (41–45). This hypoxic state activates the HIF-1 signaling pathway and its gene targets, including the angiogenic factor VEGF, which drives neovascularization during neointimal and plaque formation (40, 46). Interestingly, our findings suggest that the mechanisms of vasa vasorum remodeling in the setting of human ascending aortic aneurysm markedly differ from those observed in atherosclerosis. In our study, the presence of lymphoplasmacytic infiltration near small-diameter vessels in the adventitia of degenerative TAA might contribute to poor expansion of the vasa vasorum in these patients. This observation of an inflammatory process in the adventitia is consistent with prior work by others in cases of thoracic aortic aneurysm (47) and related to IgG4 in aortic dissection (48) though these studies did not include inspection of specimens from patients with BAV. In our study, there was no history or suspicion of arteritis in patients from which aortic specimens revealing evidence of chronic inflammation in the adventitia were obtained, thus implicating an inflammatory component in degenerative aneurysmal disease prior to, or in the absence of dissection and patients without BAV.

In the setting of ascending aortic aneurysms, we characterized vasa vasorum remodeling by a depletion of small vessels (≤ 50 μm) with an associated decrease in the pro-angiogenic factors *Hif-1*α and *Vegf-A* gene expression and increased levels of the antiangiogenic factor TSP1, together pointing to decreased angiogenic capacity. These observations are consistent with our recent work revealing decreased levels of angiogenic factors in the adventitial extracellular matrix of aneurysmal ascending aortic specimens when compared to non-aneurysmal specimens, determined utilizing an angiogenic array (49). Our data corroborate the study by Kessler et al. which reported a decrease in VEGF at the mRNA level in the adventitia of human TAA specimens and found no difference at the protein level using ELISA (50). Information on adventitial microvessel prevalence or morphometrics was not previously reported (50). Our study adds new knowledge on adventitial vasa vasorum and confirms elevated TSP1 in the adventitia of aneurysmal aorta (50). Interestingly, Kessler et al. reported increased density of microvessels in the media of aneurysmal ascending aortic specimens from patients with TAV associated with increased expression of key pro-angiogenic factors in the medial layer, such as angiopoietin-1 and -2, and FGF1 (50). Moreover, we observed wall thickening of vasa vasorum observed in our aneurysmal specimens, which could be an indication of arteriogenesis. While we can neither rule out nor confirm involvement of arteriogenesis in the observed changes in the vasa vasorum network of human TAA, possible mechanisms underlying wall thickening include microvascular shear stress and changes in fluid dynamics or pressure. Altered hemodynamics are known to occur in the aorta itself in the setting of TAA (51) but whether the vasa vasorum also experiences shear stress and changes in fluid dynamics and pressure or is affected by hemodynamic changes in the parent vessel remains unknown. Nevertheless, our observations highlight alterations in pro- and anti-angiogenic signals, and their specific impact on the vasa vasorum network in the pathophysiology of ascending aortic aneurysms warrants further study.

Based on our study and others, it appears that TAAs exhibit remodeling of vasa vasorum and dysregulation of hypoxia- and angiogenesis-related factors. These data in human aorta are supported by several earlier studies in animal models that demonstrate the importance of adventitial vasa vasorum in medial homeostasis of the host. The study by Wilens et al. in canine was the first to show a direct link between interruption of blood flow through the vasa vasorum of the descending aorta and necrosis of the aortic media (11). These observations demonstrating the importance of vasa vasorum in aortic wall homeostasis were corroborated by other investigators studying the impact of vasa vasorum occlusion in porcine and rabbit models who described medial necrosis evidenced by localized areas of SMC loss, and sparse and discontinuous elastin fibers (10, 13, 14). These histopathologic phenomena are reminiscent of the hallmarks of human TAA known as cystic medial degeneration. Although these studies did not establish a direct link between blood flow in the vasa vasorum and aneurysm development, a recent study in rat by Tanaka et al. showed that hypoperfusion of adventitial vasa vasorum led to medial hypoxia associated with aneurysmal development in the abdominal aorta (52). Determination of remodeled vessel function including endothelial-dependent vasoreactivity and NO signaling capacity and the influence of extracellular cues in the setting of aneurysmal disease could offer insights on how vasa vasorum remodeling affects media biology and biomechanics.

Whether or not vasa vasorum remodeling directly influences the risk of aneurysm and subsequent dissection in human ascending aortic aneurysms is unclear. Pursuit of this notion is supported by knowledge that human Type A aortic dissection commonly propagates in the adventitia-media border and reports of dissection alongside the vasa vasorum pathway (35). Furthermore, Niinimaki et al. found that expression level of the hypoxia marker carbonic anhydrase IX increased with the diameter of aortic aneurysms, supporting our own findings in specimens from TAV patients, where we revealed a positive correlation between Glut1 expression and ascending aortic diameter. In this same study, specimens from patients presenting with acute aortic dissection displayed carbonic anhydrase IX positive staining (29). These observations suggest a possible connection between hypoxic levels and TAA disease progression into aortic dissection. Lastly, the possible role of altered vasa vasorum in the risk of dissection is further supported by the observation of leaky neovessels and accumulation of plasma proteins in the media of TAA specimens (50). Based on these observations, Mallat et al. proposed that dysfunctional vasa vasorum may be key in the initiation of aortic dissection (53). While these observations collectively point to a possible association between vasa vasorum dysfunction in the progression of TAA toward dissection, the impact of not only microvascular remodeling and possible dysfunction but also medial and adventitial integrity in the setting of TAA deserve further consideration.

Our study revealed a few differences between aortopathy related to the presence of BAV and in patients with the morphologically normal TAV. Specifically, aneurysms in patients with TAV displayed lower vasa vasorum density when compared to that of patients with BAV, and the density of vasa vasorum was inversely related to increasing aortic diameter. Additionally, thickening of the vasa vasorum wall and locally increased GLUT1 expression were only found in aneurysmal specimens from patients with TAV. Gaining acceptance is the concept that aneurysms arising in patients with BAV are mechanistically distinct from those arising in TAV patients (21, 54), others have started to consider differences in the adventitial layer (50). Collectively, these observations add to a growing body of literature describing the distinctions in the mechanisms involved in the pathophysiology of BAV- and TAV-related TAA and could help explain why patients with BAV seem no more likely to dissect than patients with TAV (55, 56). Because we noted distinct differences in the adventitia of aortic specimens from BAV and TAV patients, we continue to pursue understanding how the extracellular cues influence cell behavior in all layers of the aortic wall.

In conclusion, we describe here several interesting anomalies in vasa vasorum size, abundance, and thickness in the setting of ascending thoracic aortic aneurysm. Wall thickening, SMC hyperplasia and lumen dilatation of the vasa vasorum are all changes that could limit nutrient delivery in the host vessel. Furthermore, our observations of down-regulated expression of angiogenic and hypoxia-related gene targets in the adventitia associated with evidence of chronic hypoxia in the media suggest a complex interplay among hypoxic signaling, microvascular function, and ascending aortic aneurysm pathophysiology. These findings have wide-spread implications for increasing our understanding of perivascular influence of vascular homeostasis and mechanisms of aortic disease.

## Limitations and future perspectives

The focus of our study on resected samples of human aorta imposes a few limitations on the extent to which our results can be interpreted. Whether the noted vasa vasorum remodeling is a cause or a consequence of the aneurysmal pathology requires further study. The subject of our ongoing work includes developing appropriate human cell and tissue-based disease models to study microvascular physiology in the setting of human aortic disease. New animal models might prove useful in deciphering mechanisms of putative microvascular dysfunction related to human aortic disease that could be distinct from mechanisms at play in the abdominal aorta. Likewise, the influence of adventitial biology on media homeostasis may be both anatomically and etiologically-specific. Inspection of vasa vasorum physiology in smaller aneurysm (< 45 mm) might offer additional insights into pathways of early disease and provide new information of what factors dictate progressive degeneration of the aortic media, leading to biomechanical failure. These areas collectively shape the focus of our ongoing trajectory toward a comprehensive multi-layer understanding of human aortic pathophysiology.

## Author contributions

MB, JH, TR, and JP participated in experimental data collection. MB and JP performed morphometric analyses, while qPCR data were analyzed by JH. MB completed all additional analyses. MB and JP generated the manuscript with input from TG. JP supervised the entire study.

### Conflict of interest statement

The authors declare that the research was conducted in the absence of any commercial or financial relationships that could be construed as a potential conflict of interest.
